# Distributed Cluster Regulation Strategy of Multipark Integrated Energy System Using Multilayer Deep Q Learning

**DOI:** 10.1155/2022/5151369

**Published:** 2022-10-12

**Authors:** Chaoqun Zhu, Jie Shen, Jie Li, Xiaoming Zhang, Lei Zhou, Dan Zhu, Yafei Li

**Affiliations:** State Grid Corporation of China, Marketing Department of Suzhou Branch, Suzhou 215000, China

## Abstract

The power system is evolving from a single energy system to an integrated energy system. In order to further improve the power generation and consumption balance capacity of the park integrated energy system (PIES), the park integrated energy system is gradually transitioning from the single park energy system operation mode to the multipark energy system operation mode. The design of multipark integrated energy system (MPIES) collaborative control strategy will become an important part to improve the power generation and consumption balance ability of the integrated energy system. In order to fully tap the regulation capacity of each PIES, we propose a coordinated control strategy for the integrated energy system in multiple parks considering the flexible substitution interval of multiple types of energy. Firstly, we analyze the influence of the types of regulation resources and the regulation incentive mechanism of the PIES on the regulation flexible range of the PIES. Then, based on the Markov decision process, a distributed cluster regulation model of MPIES considering regulation demand and regulation flexible interval is established. Finally, using multilayer deep Q networks (MLDQN), the distributed cluster regulation optimization algorithm of MPIES is given. The simulation results show that the proposed method can coordinate the regulation ability of each park integrated energy system in the MPIES, give full play to the large-scale advantage of the interconnection of the park integrated energy system, and improve the overall stability of the multipark integrated energy system.

## 1. Introduction

The flexibility and security requirements of the society for energy demand are constantly improving, which makes the traditional centralized large-scale power system change to the distributed integrated energy system [1]. The development of combined heat and power plants, gas turbines, and other multienergy conversion technologies is accelerating the transformation of the energy structure [2, 3]. Park integrated energy system has become a bearing platform for efficient utilization of clean energy [4]. The flexible resources in the integrated energy system of a single park have high uncertainty, and the combination of multiple PIES can realize the complementary coordination of different parks and different energy sources and reduce the overall uncertainty. With the goal of improving system economy, safety, reliability, and environmental protection, flexibly adjusting MPIES operation mode and promoting the safe consumption of clean energy in the power grid has become a research hotspot in academia and industry in recent years.

The park integrated energy system achieves the cross-energy response of power system demand through energy coupling equipment [5–7]. In the regulation process, it is necessary to balance the relationship between the economy and security of the park integrated energy system, and comprehensively consider the operation status of subsystems and the overall operation status of the system. In Reference [8], a multiobjective optimization model for the design of integrated electric, thermal, and cooling energy system is established from the aspects of economy and environment, and the selection and configuration of various components of the system are carried out. In Reference [9], PIES is divided into three modules for analysis based on hub model, and a PIES day ahead optimal scheduling model is established considering the economy target and security constraints. Reference [10] points out that the static programming strategy of PIES reduces the economy and reliability of the system. A two-stage robust model is proposed to reduce the impact of uncertainty in PIES. To solve the optimization model, the column and constraint generation algorithm is adopted. Reference [11] studies the risks brought by the uncertainty of natural gas price and electricity price to PIES planning and establishes a PIES planning risk assessment model considering the uncertainty of energy price. Conditional value-at-risk is used as a risk index to quantify the impact of uncertainty on PIES planning. When evaluating the benefits of an integrated energy system, because the selected benefit evaluation indicators are incomplete, the expected benefit evaluation results are distorted, resulting in large economic losses. Therefore, many scholars have conducted in-depth research on benefit evaluation index information and benefit evaluation methods [12–15]. Reference [16] proposes a distributed energy system evaluation index system from the four dimensions of technology, economy, environment, and society and used the principle of maximum entropy and an improved grey correlation method to evaluate the benefits of integrated energy systems. These studies have laid a foundation for the study of the coordinated regulation of the park integrated energy system.

The multiobjective optimization solution of the park integrated energy system has an important impact on the collaborative optimization of the integrated energy system [17–19]. Reference [20] establishes a multiobjective optimization model for building integrated energy system and solves the above model by analytical method and heuristic method. According to the operation structure of energy storage device, electrothermal conversion equipment, and demand response mechanism, the authors in Reference [21] establish a multiobjective model of electric thermal water energy system by introducing user comfort and solving it by using integer programming theory. Reference [22] adopts the multiobjective optimization model generation scheme and portfolio constraint method to solve the multiobjective optimization model of urban integrated energy system. For the large-scale renewable energy access operation system, Bravo et al. [23] designed a hybrid solar power plant considering thermochemical energy storage devices, established the corresponding multiobjective optimization model, and used the multiobjective solution method to solve it.

Reinforcement learning can effectively solve the optimal scheduling problem. In Reference [24], an optimal scheduling model based on automated reinforcement learning is proposed to address the error accumulation issue. Authors in Reference [25] introduce the reinforcement learning model to solve the charging station optimal scheduling problem. It can be learned that the reinforcement learning model can be used to compensate for the resource requirements mismatch on the energy scale. In Reference [26], the authors define energy storage systems usage standards for an adaptive power transaction plan based on reinforcement learning. The author decomposes the life cycle cost into four variables to make the model meet the model requirements of reinforcement learning. It can be seen that in the reinforcement learning framework, the optimal scheduling problem can be effectively solved.

Although the current research has made a lot of research results in the field of park integrated energy coordinated regulation strategy, there are still deficiencies in the following aspects:

1. When analyzing the regulation capacity of the park integrated energy system, the impact of resource types, subsidy policies, and time changes on the regulation flexibility range in the park integrated energy system were not comprehensively considered.
2. When studying the coordinated regulation strategy of multipark integrated energy system, the influence of the flexible regulation range of the integrated energy system in the lower park on the allocation of regulation tasks by the upper regulation center was not considered.

In view of the above problems, this paper proposes a distributed cluster regulation strategy of multipark integrated energy system considering the regulation of flexible intervals. This paper analyzes the regulation demand of multipark integrated energy system, the time cost attribute of flexible regulation resources, and the demand regulation task allocation method considering the regulation flexible interval. The multilayer deep Q network is used to realize the coordinated regulation of multipark integrated energy system, reduce the regulation pressure under the typical problem scenario of multipark integrated energy system, and give play to the interconnection advantage of multipark integrated energy system.

The main contributions of the paper are three-fold, which are as follows:

1. The flexible range of the regulation ability of the flexible resources in PIES under the time scale is analyzed, which provides the basis for formulating the timing regulation instructions of PIES.
2. The decision-making method of flexible interval allocation of regulation tasks by the upper control center combined with the regulation ability of the lower PIES is studied.
3. Under the reinforcement learning framework, the regulation state and decision-making behavior models of upper MPIES and lower PIES are established, and a two-level regulation optimization model considering the flexible range of PIES regulation is realized. On this basis, the multilayer deep Q network is used to realize the optimization solution method of the MPIES double-layer collaborative regulation strategy.

The scope of the paper is shown as follows: first, the two-level coordinated regulation model of MPIES is discussed in this paper; then, the cooperative regulation strategy of MPIES considering the regulation flexible interval is studied; finally, the optimization algorithm of the proposed MPIES regulation model is proposed based on multilayer deep Q network.

The remaining parts of the paper are organized as follows: in Section 2, the two-level coordinated regulation model of MPIES is discussed. In Section 3, the cooperative regulation strategy of MPIES considering the regulation flexible interval is studied. In Section 4, the optimization algorithm of the proposed MPIES regulation model is proposed based on multilayer deep Q network. In Section 5, simulation results are carried out to verify the proposed regulation strategy. Finally, Section 6 states conclusions.

## 2. Two-Level Coordinated Regulation Model of MPIES

### 2.1. Basis of MPIES Regulation Model

As shown in Figure 1, the MPIES double-layer collaborative regulation model studied in this paper is mainly composed of the upper control center and multipark integrated energy systems. The PIES includes electric energy system, thermal energy system, and gas system. Each energy system has resources that can be flexibly adjusted, and each energy system can use energy conversion equipment to realize energy substitution. The flexibility of the integrated energy system is mainly reflected in the following two aspects:

  Energy convertibility: compared with the previous independent energy supply subsystems divided by energy types, the advantage of the integrated energy system is that it can break the independent state of each energy subsystem to realize multienergy coupling and cross-energy supply, and each energy subsystem can be regarded as a whole. In order to achieve overall management and collaborative optimization, the integrated energy system couples and associates different energy flow paths through conversion equipment. Compared with the traditional independent energy flow system, it provides more redundant energy flow conversion paths and provides more space for multienergy system optimization. For example, for thermal energy, gas can be converted into heat by the combined equipment of combined heat and power (CHP) unit and waste heat exchanger, electricity can be converted into heat by electric furnace, and gas can be directly converted into heat by gas boiler. On the grid source side, due to the existence of energy conversion equipment such as CHP units and electric heating furnaces, the energy flow is convertible. For thermal energy, it can be converted to heat by gas or electricity.
  Energy substitutability: in terms of energy consumption, users have room to choose among different energy flows, that is, there are alternatives among energy flows for energy supply when the load is used. If a load can choose two or more energy flows and can meet its own load requirements, it means that the load is replaceable, which is called a substitute load. The more energy types a load can choose from and the larger the capacity of the load-side consumer equipment, the higher the substitutability of the load, which means that the user has more choices. Generally speaking, the load of the integrated energy system can be divided into four categories: cooling load, heat load, electrical load, and gas load. Here, the heat load is used as an example to illustrate the substitutability of the load. If the user can freely choose heating network heating (such as central heating), grid heating (such as electric water heater), gas network heating (such as gas water heater), and other methods to meet the heat demand, and the energy consumption of each method is also with selectivity, it means that the heat load has certain substitutability.

The above two characteristics of the integrated energy system provide the basis for the coordinated regulation of multi-PIESs.

In the process of MPIES regulation, the lower-level PIES will upload the operation status information of the energy systems in the area under their jurisdiction to the upper-level regulation center. According to the overall regulation objectives of the current MPIES, the upper-level control center considers the regulation uncertainty interval of each PIES, formulates an effective and economic regulation plan, and issues it to each control center of PIES. According to the overall task issued by the upper control center, the lower-level PIES disassembles the overall regulation task with the minimum cost on the premise of ensuring the completion of the regulation task, combined with the flexible range of regulation resources in the region under its jurisdiction. The disassembled adjustment task will be allocated to various types of flexible resources for adjustment.

### 2.2. Flexibility Analysis of Regulating Resources in PIES

In the process of regulation, the regulation ability of various types of regulatory resources in PIES will show dynamic characteristics with the change of time. The regulating ability of regulating resources at the current time is affected by both the current time and the historical time. Accordingly, the regulation behavior of flexible resources at the current time will also affect the regulation ability in the future time. In order to record the cumulative changes of the flexible interval of regulation resources over time, this paper defines the cumulative regulation state of regulation resources in PIES, which is given below:

(1) $$\begin{array}{c} F_{i,t}^{s}=\int_{0}^{t}a_{i,t}^{s}dt\text{.} \end{array}$$

It can be seen that *F*_*i*,*t*_^*s*^ can represent the change in the adjustment range of flexible resources in the remaining period, thus affecting the formulation of adjustment instructions at the current time.

At the same time, the subsidy strategy for regulating resources will also affect the regulation flexibility range of flexible resources in PIES. When the adjustment subsidy for flexible resources reaches a certain amount, users in PIES will be willing to respond to the upper-level control instructions by changing the energy consumption mode. This paper establishes a model of the flexible range of PIES flexible resources and subsidy strategy, as given below:

(2) $$\begin{array}{c} G_{i,t}^{ra}\left(s_{i,t}^{ra}\right)=\left\{\begin{array}{c} 0,s_{i,t}^{ra}<s_{i,t}^{\text{low}},\\ \eta^{ra}\;\ln\;\left(s_{i,t}^{ra}-s_{i,t}^{\text{low}}+\varepsilon \right),s_{i,t}^{\text{low}}\leq s_{i,t}^{ra}\leq s_{i,t}^{\text{up}} \end{array}\right.\text{.} \end{array}$$

When the subsidy amount *s*_*i*,*t*_^*ra*^ for the regulated resources is less than the minimum subsidy amount *s*_*i*,*t*_^low^ that the flexible resource subject is willing to participate in the regulation, the flexible resource regulated resources in PIES are 0. When *s*_*i*,*t*_^*ra*^ ≥ *s*_*i*,*t*_^low^, the flexible resource subject will adjust its flexible adjustment ability according to the subsidy amount. The model of subsidy cost is given below:

(3) $$\begin{array}{c} C_{i,t}^{s}=f\left(s_{i,t}^{ra},p_{i,t}^{gr},a_{i,t}^{s}\right)\text{.} \end{array}$$

## 3. Cooperative Regulation Strategy of MPIES Considering the Regulation Flexible Interval

### 3.1. Collaborative Regulation Task Allocation Mechanism

For PIES-*i* in MPIES, at time *t*, its adjustment flexibility interval *R*_*i*,*t*_^*r*^ can be expressed as given below:

(4) $$\begin{array}{c} R_{i,t}^{r}=\left\{\begin{array}{c} R_{i,t}^{r,\text{up}}-R_{i,t}^{r,\text{low}},\\ \begin{array}{c} R_{i,t}^{r,\text{up}}=S_{i,t}^{\text{cut},u}+S_{i,t}^{\text{swift},u}+S_{i,t}^{es,d},\\ R_{i,t}^{r,\text{low}}=S_{i,t}^{\text{cut},l}+S_{i,t}^{\text{swift},l}+S_{i,t}^{es,c}, \end{array} \end{array}\right. \end{array}$$

The regulation plan of PIES-*i* in regulation cycle *k* can be expressed as given below:

(5) $$\begin{array}{c} Sh_{i,t}=Sh_{i,t}^{\text{up}}\frac{R_{i,t}^{r}}{\overset{n_{mg}}{\underset{i=1}{\sum }}R_{i,t}^{r}}\text{.} \end{array}$$

Considering the problems of exploration and utilization, reward sparseness, and local optimization that may exist in the decision-making process, compared with completely random assignment of peak shaving tasks, the scheduling control center considers the peak shaving task allocation decision made by the state information of the elastic amplitude of each region at the current moment, and further. Using the system elastic resource information, the local optimum can be avoided to a certain extent. Use the elastic range to guide the assignment of peak shaving tasks, take a more logical and realistic initial assignment task as a starting point, and then carry out learning optimization and correction, to a certain extent, more optimal (or suboptimal) peak shaving can be obtained. In addition, the comprehensive energy system of the park with large flexibility has a larger peak-to-valley electricity price difference. Combined with the time-of-use electricity price, it is more conducive to peak shaving and valley filling and stable and economic operation of the system.

### 3.2. Regulation Model Based on Markov Process

#### 3.2.1. Control Center Optimization Model of MPIES

In this section, a regulation cycle is divided into *k* decision cycles. The state *s*_*k*_^*cl*^ of the control center of MPIES at the decision-making time *t*_*k*_ can be expressed as given below:

(6) $$\begin{array}{c} s_{k}^{cl}=\left(t_{k},r_{k}^{\text{task}},s_{k}^{e,1},s_{k}^{e,2},s_{k}^{e,i},s_{k}^{e,n_{mg}}\right)\text{.} \end{array}$$

Let *s*_total_^*cl*^ be the state space of the control center of the MPIES, then there is *s*_*k*_^*cl*^ ∈ *s*_total_^*cl*^. The number of states of MPIES can be expressed as given below:

(7) $$\begin{array}{c} n_{s}^{\max}=T^{t}\left(n_{\text{task}}+1\right)\overset{N}{\underset{i=1}{\prod }}\left[\left(2n_{i}^{es}+1\right)\left(2n_{i}^{\text{swift}}+1\right)\left(2n_{i}^{R}+1\right)\right]\text{.} \end{array}$$

At time *t*, the control task assigned by the control center of MPIES to PIES *i* is as follows:

(8) $$\begin{array}{c} C_{i,t}^{\text{task}}=\frac{P_{t}^{\max}}{n^{\text{dis}}}a_{i,t}^{mg}\text{.} \end{array}$$

*a*_*i*,*t*_^*mg*^ is the task allocation behavior of the MPIES to PIES *i* at time *t*, and satisfies the expression, which is given below:

(9) $$\begin{array}{c} \overset{n_{mg}}{\underset{i=1}{\sum }}a_{i,t}^{mg}=n^{\text{dis}}\text{.} \end{array}$$

For the MPIES, the evolution process of the regulation model can be controlled by task allocation behavior *a*_*i*,*t*_^*mg*^=*S*_str_^*cl*^(*s*_*t*_^*cl*^) based on the decision strategy *S*_str_^*cl*^ in combination with the state *s*_*t*_^*cl*^ of time *t*.

The operation cost *C*_*k*_^*cl*^ of the MPIES at the decision-making time *t* is set as the superposition of the operation costs of each PIES, specifically:

(10) $$\begin{array}{c} C_{k}^{cl}=\overset{n_{mg}}{\underset{i=1}{\sum }}C_{i,k}^{mg}\text{.} \end{array}$$

On the other hand, considering the multiperiodicity of the regulation of MPIES, that is, the regulation strategy tends to make the regulation capacity of the energy storage device in the initial state of the regulation cycle and the transferable load as consistent as possible with the end state of the regulation cycle, so as to provide sufficient regulation resources for the next regulation cycle. Therefore, this paper further considers the transfer cost of flexible resource regulation capability. The transfer cost of flexible resource regulation capability of MPIES is expressed as the sum of the transfer cost of each PIES energy storage device (*C*_*i*,*k*_^*es*^) and the transfer cost of transferable load (*C*_*i*,*k*_^*sw*^).

For the MPIES control center, under strategy *S*_str_^*cl*^, the optimization performance criterion with the initial state of *s*_0_^sta^ is _*I*_^strup^, then there is

(11) $$\begin{array}{c} {}_{I}^{\text{strup}}=E_{\text{str},0}^{\text{up}}\left[\overset{K-1}{\underset{k=0}{\sum }}c_{k}^{cl}+\overset{n_{mg}}{\underset{i=1}{\sum }}C_{i,k}^{es}+\overset{n_{mg}}{\underset{i=1}{\sum }}C_{i,k}^{sw}\right]\text{.} \end{array}$$

Then the optimization objective of the MPIES control center can be expressed as given below:

(12) $$\begin{array}{c} S_{\text{str}}^{cl,o}=arg\;\;\min{}_{I}^{\text{strup}}\text{.} \end{array}$$

That is, the optimization goal of the MPIES is to find the optimal strategy in the available strategy set of the MPIES control center so that the overall operation cost of the MPIES is the lowest, and the regulation capacity of the energy storage device and the transferable load at the end of the regulation cycle is restored to the initial level as far as possible.

#### 3.2.2. Regulation Model of PIES

Similar to the state of MPIES, the state *s*_*k*_^*mg*^ of PIES *i* at decision time *t* can be expressed as given below:

(13) $$\begin{array}{c} s_{k}^{mg,i}=\left(t_{k},l_{k}^{\text{task},i},s_{k}^{e,i}\right)\text{.} \end{array}$$

Let *s*_total_^*mg*,*i*^ be the state space of PIES *i*, then there is*s*_*k*_^*mg*,*i*^ ∈ *s*_total_^*mg*,*i*^. The number of states *n*_*mg*,*i*_^max^ of the PIES can be expressed as given below:

(14) $$\begin{array}{c} n_{mg,i}^{\max}=kn^{\text{dis}}\left(2n_{i}^{es}+1\right)\left(2n_{i}^{\text{swift}}+1\right)\text{.} \end{array}$$

The action *a*_*i*,*t*_^*un*^ of PIES *i* at time *t* consists of the action of energy storage system *a*_*i*,*k*_^*es*^, the action of flexible resources *a*_*i*,*k*_^*fr*^ and the action of subsidy strategy *a*_*i*,*k*_^*re*^. *a*_*i*,*t*_^*un*^ can be written as follows:

(15) $$\begin{array}{c} a_{i,k}^{un}=\left(a_{i,k}^{es},a_{i,k}^{fr},a_{i,k}^{re}\right)\text{,} \end{array}$$

where the regulation methods of the energy storage device include discharge, standby, and charging; The adjustment methods of flexible resources include reduction action and transfer action; The subsidy strategy includes a variety of optional subsidy amounts.

## 4. Optimization Algorithm of the Two-Level MPIES Regulation Model

Each PIES in the MPIES has a variety of flexible resources that can be used to participate in regulation. Accordingly, the PIES state action set composed of the states and actions of these flexible resources presents a large-scale feature. For the MPIES control center, these PIESs with large-scale state action sets will bring more complex matrix dimensions to the overall control model of the MPIES. To solve this problem, this paper constructs the optimization solution model of MPIES regulation model based on multilayer deep Q network.

The interaction model of MPIES regulation is shown in Figure 2. Based on the status and regulation demand of each PIES in the current system, the MPIES selects the decision-making behavior in the decision-making behavior set and sends the regulation instructions to each PIES. After obtaining the overall regulation instructions of the PIES allocated, each PIES will split the regulation instructions into specific regulation resources in combination with the regulation ability of its own various regulation resources and summarize the decision rewards in this round of decision-making cycle to the MPIES to form the overall decision rewards of the MPIES, so as to guide the decision-making behavior of the next decision-making cycle.

The specific steps of optimizing the regulation model of MPIES based on multilayer deep Q network are as follows:

  Step 1. Initialize the parameters of the MPIES model. It mainly includes the number of decision-making cycles, the number of discrete levels of MPIES regulation, the number of discrete levels of maximum power of each PIES energy storage system, the number of discrete levels of maximum power that can reduce the load, the electricity price in the decision-making cycle, and the flexible range of each PIES regulation.
  Step 2. Initialize the depth Q network parameters. Including various parameters of Q network, PIES group, and Q value table of each PIES.
  Step 3. Select the regulation behavior from the MPIES decision-making behavior set and distribute it to each PIES.
  Step 4. Select the regulation behavior from the decision behavior set of each PIES and distribute it to each regulation resource to form the decision reward of each PIES in the current decision cycle and summarize it to the regulation center of the MPIES.
  Step 5. Update the Q value table of each PIES.
  Step 6. Update the Q value table of MPIES.
  Step 7. If the decision-making process is not completed, return to step 3; If the decision-making process is completed, the optimization decision-making process ends.

The flowchart of the optimization model is shown in Figure 3.

## 5. Simulations and Analysis

The Simulation considered in this section is: the MPIES composed of three PIESs performs collaborative peak shaving in the intraday scenario. It is considered that the daily scheduling cycle is divided into 24 decision-making periods.

Among the loads of PIES1, the load that cannot be flexibly converted accounts for about 85.3%, and the load that can be flexibly converted accounts for about 14.7%, of which the load that can be reduced and the load that can be transferred account for 9% and 5.7%, respectively. In PIES2 and PIES3, the load that cannot be flexibly converted accounts for about 85%, and the load that can be flexibly converted accounts for about 15%. The capacity of VRB energy storage devices equipped in different areas is as follows: PIES1 has 6MWh energy storage, PIES2 has 5MWh energy storage, and PIES3 has 3MWh energy storage. The overall regulation instructions of the MPIES control center are shown in Figure 4.

Figure 5 shows the load curve of the MPIES based on the collaborative optimization strategy proposed in this paper. The peak valley difference of the overall load of the MPIES before optimization is large, reaching 6481 kW. The coordinated regulation strategy of MPIES based on multilayer deep Q network regulates the flexible resources in the MPIES as a whole so that the fluctuation of the overall power load in the MPIES tends to be stable, and the intraday peak valley difference is reduced to 2513 kW, which greatly reduces the peak regulation pressure of the MPIES.

Figure 6 shows the proportion of peak shaving time and peak shaving volume of flexible resources of each PIES in the MPIES before and after optimization, respectively. It can be seen that before optimization, the MPIES control center assigned more control tasks to PIES 1, whereas PIES 3 was only assigned less control tasks. This allocation result is determined by the flexible resource characteristics of each PIES. When the regulation center of the MPIES tends to consider the PIES with stable and flexible resources first (such as PIES 1), it will directly assign more regulation tasks to it, and there is a possibility that the flexible resources of the current PIES may be exhausted in a certain period of time. The collaborative regulation strategy of MPIES considering flexible interval proposed in this paper comprehensively considers the flexible interval of flexible resources of each PIES in the MPIES, searches for the optimal allocation behavior under the overall flexible interval and can dynamically update the allocation behavior according to the iterated state of the MPIES, so as to activate the potential of flexible resources with uncertainty. The stable and flexible resources are partially released from a single implementation and regulation task to improve the stability of the overall regulation of the MPIES.

Figures 7–9 show the decision-making behavior of each PIES in each period of the dispatching day. Among them, the blue histogram cut indicates the resources that can be flexibly reduced, and when it is greater than zero, it indicates that the reduction behavior of the corresponding instructions is executed. The orange histogram swift indicates the flexible resources that can be transferred in the time series. When it is greater than zero, it indicates the reduction behavior of the corresponding instructions, and when it is less than zero, it is the recovery behavior. The grey histogram energy store indicates the behavior of the energy storage device. When it is greater than zero, it indicates the discharge behavior, and when it is less than zero, it indicates the charging behavior. Each PIES calls flexible resources in the PIES based on the task collaborative allocation instruction of the control center of the MPIES.

Figure 7 shows the action selection of PIES 1 in each period under the optimization strategy. For the resources that can be flexibly reduced, the reduction action will not be taken during the low power consumption period. In the period of demand for reduction, the total load of the current PIES will be reduced in accordance with the overall regulation task of the PIES and with the transfer of flexible resources and energy storage devices. There will be a large reduction during the peak period of power consumption. For transferable flexible resources, they will cooperate with other types of flexible resources to reduce during some peak periods of power consumption, but usually, the adjustment amount is not large, because it is necessary to arrange transferable flexible resources to restore during the peak period of power consumption. The regulation characteristics of the energy storage device are similar to the regulation characteristics of flexible resources that can be transferred. It will discharge during the peak period of power consumption and charge during the low period of power consumption with low electricity price.

Figures 8 and 9 show the regulation behavior of flexible resources in PIES 2 and PIES 3. Compared with the regulation behavior of each flexible resource in PIES 1 shown in Figure 6, the flexible resources under PIES 2 and 3 participate in the overall peak shaving task of the MPIES to a certain extent. Although the overall regulation is smaller than that generated by the flexible resources of PIES 1, it can still play an important role in regulation. Considering the high uncertainty of flexible resources in PIES 3, part of the regulation actions of PIES 1 and PIES 2 are used to make up for the uncertainty of flexible resources in PIES 3 in the process of MPIES coordination, which makes PIES 1 and PIES 2 call more energy storage devices than PIES 3, thereby increasing the stability of the overall regulation of MPIES.

## 6. Conclusion

This paper studies the distributed cluster regulation technology of MPIES considering the flexible interval of regulation resources. First, the flexible range of the regulation capability of the flexible resources in the PIES under the time scale is analyzed, which provides a basis for formulating the PIES time sequence regulation instructions. Then, the decision-making method of the upper-layer MPIES controller combined with the regulation ability of each lower-layer PIES to allocate regulation tasks flexibly is studied. Finally, under the framework of reinforcement learning, the regulation status and decision-making behavior models of the upper-layer MPIES and the lower-layer PIES are established, and a two-layer regulation optimization model considering the flexible range of PIES regulation is realized. On this basis, a multilayer deep Q network is used to realize the optimal solution method of the two-layer coordinated regulation strategy of the MPIES. The simulation results show that the two-layer coordinated regulation architecture of the MPIES proposed in this paper has good regulation performance.

From the perspective of practical application, although the algorithm proposed in this paper has good solution performance, the convergence of optimization solution is difficult, and it is difficult to obtain the optimal solution in some scenarios. In the following research, it is necessary to consider appropriately relaxing some constraints on variables to make the model robust.

## Figures and Tables

**Figure 1:** Schematic diagram of MPIES hierarchical collaborative regulation structure.

**Figure 2:** Schematic diagram of interaction between upper and lower levels in the process of scheduling optimization.

**Figure 3:** Flowchart of the optimization model.

**Figure 4:** Peak shaving demand curve of MPIES.

**Figure 5:** Collaborative optimization curve of load in MPIES.

**Figure 6:** Peak shaving of PIES before and after optimization. (a) Proportion of peak shaving time before optimization, (b) proportion of peak shaving time after optimization, (c) Proportion of peak shaving before optimization, and (d) Proportion of peak shaving after optimization.

**Figure 7:** Action selection of PIES 1 in each period under the optimization strategy.

**Figure 8:** Action selection of PIES 2 in each period under the optimization strategy.

**Figure 9:** Action selection of PIES 3 in each period under the optimization strategy.

## Data Availability

The data used to support the findings of this study can be obtained from the corresponding author upon request.

## Indices and variables:

*a*_*i*,*t*_^*s*^: Actual demand state of PIES
*F*_*i*,*t*_^*s*^: Adjustment ability of flexible resources
*G*_*i*,*t*_^*ra*^: Flexible adjustment capability of PIES
*s*_*i*,*t*_^*ra*^: Subsidy amount for the regulated resources
*s*_*i*,*t*_^low^: Minimum subsidy amount
*η* ^*ra*^: Subsidy-response coefficient; *ε* Constant number for calculating *G*_*i*,*t*_^*ra*^
*p*_*i*,*t*_^*gr*^: Time of use price of PIES
*R*_*i*,*t*_^*r*,up^: Upper bounds of the flexible range
*R*_*i*,*t*_^*r*,low^: Lower bounds of the flexible range
*S*_*i*,*t*_^cut,*u*^: Upper bounds of resources that can be reduced
*S*_*i*,*t*_^cut,*l*^: Lower bounds of resources that can be reduced
*S*_*i*,*t*_^swift,*u*^: Upper bounds of transferable resources
*S*_*i*,*t*_^swift,*l*^: Lower bounds of transferable resources
*S*_*i*,*t*_^*es*,*d*^: Discharge margin of energy storage device
*S*_*i*,*t*_^*es*,*c*^: Charge margin of energy storage device
*n*_*mg*_: Number of PIES in MPIES
*i*: Index of PIES
*t*: Regulation time
*r*_*k*_^task^: Real-time adjustment demand
*s*_*k*_^*e*,*i*^: System status information of PIES
*P*_*t*_^max^: Maximum regulation demand of the MPIES
*n* ^dis^: Discrete quantity of the maximum demand
CHP: Combined heat and power
PIES: Park integrated energy system
